# Chikusetsu saponin IVa ameliorates high fat diet-induced inflammation in adipose tissue of mice through inhibition of NLRP3 inflammasome activation and NF-κB signaling

**DOI:** 10.18632/oncotarget.16052

**Published:** 2017-03-09

**Authors:** Chengfu Yuan, Chaoqi Liu, Ting Wang, Yumin He, Zhiyong Zhou, Yaoyan Dun, Haixia Zhao, Dongming Ren, Junjie Wang, Changcheng Zhang, Ding Yuan

**Affiliations:** ^1^ College of Medical Science, China Three Gorges University, Yichang, HuBei 443002, China; ^2^ Renhe Hospital of China Three Gorges University, Yichang, HuBei 443002, China

**Keywords:** chikusetsu saponin IVa, adipose tissue inflammation, NLRP3 inflammasome, NF-κB signaling, ASC pyroptosome

## Abstract

Chronic metabolic inflammation in adipose tissue plays an important role in the development of obesity-associated diseases. Our previous study indicated that total saponins of *Panax japonicus* (SPJ) rhizoma and Chikusetsu saponin V, one main component of SPJ, could exert the anti-oxidative and anti-inflammatory effects. The present study aimed to investigate the *in vivo* and *Ex vivo* anti-inflammatory activities of another main component of SPJ, namely Chikusetsu saponin IVa (CS). CS could significantly inhibited HFD-induced lipid homeostasis, and inhibited inflammation in adipose tissue, as reflected by the decreased mRNA expression levels of inflammation-related genes and secretion of the chemokines/cytokines, inhibited the accumulation of adipose tissue macrophages (ATMs) and shifted their polarization from M1 to M2, suppressed HFD-induced expression of NLRP3 inflammasome component genes and decreased IL-1β and Caspase-1 production in mice. Moreover, CS treatment also inhibited the activation of NLRP3 inflammasome in bone marrow-derived macrophages (BMDMs). Meanwhile, CS treatment inhibited an NLRP3-induced ASC pyroptosome formation and lipopolysaccharide (LPS)-induced pyroptosis. Furthermore, CS treatment suppressed HFD-induced NF-κB signaling *in vivo* and LPS-induced NF-κB activation as reflected by the fact that their phosphorylated forms and the ratios of pNF-κB/NF-κB, pIKK/IKK, and pIκB/IκB were all decreased in EAT from HFD-fed mice treated with CS as compared with those of HFD mice. Taking together, this study has revealed that CS effectively inhibits HFD-induced inflammation in adipose tissue of mice through inhibiting both NLRP3 inflammasome activation and NF-κB signaling. Thus, CS can serve as a potential therapeutic drug in the prevention and treatment of inflammation-associated diseases.

## INTRODUCTION

Obesity is the worldwide health problem, which can increase the risk of many other chronic diseases, such as insulin resistance, type 2 diabetes, hypertension, hyperlipemia, and cardiovascular disease [1]. Obesity is also closely related with the metabolic inflammation, especially in adipose tissue [2, 3], an important organ that regulates the energy homeostasis of the whole-body. Adipocytes can secret inflammation-associated adipokines besides acting as the storage pool of excessive fat [4]. During the development of inflammation-associated diseases, several the pathological events take place, which include (a) the infiltration of bone marrow-derived macrophages (BMDMs) in adipose tissue, (b) accumulation of “crown like structures(CLS)”, (c) increased expression of pro-inflammatory genes and (d) secretion of inflammation-associated cytokines/chemokines, such as TNF-α, IL-1β, SAA3, MCP-1, IL-6, CCL-5, CXCL-1, and caspase-1 [5]. Chronic metabolic inflammation in adipose tissue plays an important role in the development of obesity-related diseases. Therefore, to ameliorate metabolic inflammation in adipose tissue can be an important way for the prevention and cure of obesity-related diseases.

The important pro-inflammatory cytokines, such as interleukine-1β (IL-1β), are involved in several kinds of inflammatory diseases [6]. Generally, for IL-1β, its production needs two steps: the first step is an NF-κB-dependent priming step, in which the transcription of pro-IL-1β and nucleotide-binding domain, leucine-rich-containing family, pyrin domain-containing-3 and/or Nod-like receptor protein 3 (NLPR3) are induced; the second step is an activation step that induces the activation of caspase-1, which can proteolytically process pro-IL-1β into biologically active IL-1β[6].

NLRP3 inflammasome is composed of several proteins, including NLRP3, caspase-1, and transient receptor potential vanilloid 4(TRPV4), which is important for the production of caspase-1 and IL-1β [7, 8]. NLRP3 inflammasome can be activated by nigericin, ATP, and monosodium urate (MSU) [7]. However, excessive activation can lead to the development of several inflammatory diseases [9]. On the other hand, the genetic ablation of NLRP3 or caspase-1 and the other components of NLRP3 inflammasome has been found to decrease IL-1β level in adipose tissue and protect against the inflammation induced by obesity [10–12]. All of these studies have indicated that the abnormal activation of NLRP3 inflammasome is tightly correlated with inflammatory diseases, although normal NLRP3 inflammasome activation can contribute to the defense of the body [9]. Therefore, to find out the agents that can selectively inhibit activation of NLRP3 inflammasome will be highly significant for prevention and treatment of inflammation-related diseases.

A number of studies have reported that some medicinal plants and their extracts, such as genistein [13], kaempferol and daidzein [14], quercetin [15] and green tea [16], possess the anti-inflammatory effects. *Panax japonicas* (PJ) is a plant belonging to family *Araliaceae Panax*, and grows in Japan and southwest of China. PJ rhizoma has been known as “the king of herbal medicine” in traditional Tujia and Hmong people in China, and used as the substitute for Ginseng roots in minority ethnic group. Recent studies have revealed that saponins, polysaccharides, volatile oil and amine acids are the main components of PJ rhizoma, and proven that they have extensive pharmacological effects [17]. Saponins of *Panax japonicus* rhizoma (SPJR), the most abundant components of PJ rhizoma, mainly contain Chikusetsu saponin V, Chikusetsu saponin IV, Chikusetsu saponin IVa (CS), Panax saponin Re, and Pjs-2 etc. [17]. In our previous studies, we had demonstrated that SPJ exerted the potent inhibitory effects on oxidation and inflammation [17, 18]. Our recent study also has revealed that Chikusetsu saponin V, one main component of SPJ, exerts the anti-inflammatory effects on acute liver injury in mice [19]. However, whether Chikusetsu saponin IVa (CS), another main component of SPJ, can have anti-inflammatory activities or can inhibit NLRP3 inflammasome remains to be determined.

Therefore, the present study aimed to investigate whether CS possesses anti-inflammatory activities or inhibitory activities on NLRP3 inflammasome. Our results demonstrated that CS could potentially improve HFD-induced lipid homeostasis and inhibit inflammation in adipose tissue of mice. *Ex vivo* and *in vivo* analyses revealed that CS could inhibit HFD-induced caspase-1 and IL-1β production from epididymal adipose tissue (EAT); CS could also inhibit the accumulation of adipose tissue macrophages (ATMs) and alter their polarization from M1 to M2. CS was capable of inhibiting both NLRP3 inflammasome activation and NF-κB signaling. This study has revealed that CS can be potentially used to prevent or cure inflammation-related diseases.

## RESULTS

### CS treatment improved HFD-induced lipid homeostasis in mice

To determine the influence of CS on HFD-induced inflammation in adipose tissue, 5-week old male mice were fed with ND, HFD, HFD+CS-L or HFD+CS-H for 16 weeks, respectively. No significant difference in food intake was seen among mice in all four groups (Supplementary Figure 1). The levels of cholesterol and triglyceride in serum and liver were increased significantly in HFD group as compared to those in ND group, whereas treatment with CS-L (50 mg/kg) and CS-H (100 mg/kg) significantly reduced HFD-induced increases in levels of both cholesterol and triglyceride (Figure 1C and 1D). These data indicate that CS can improve HFD-induced lipid homeostasis in serum and liver of mice.

**Figure 1:** CS treatment improves high fat diet-induced lipid homeostasis in mice (**A**) The chemical structure of Chikusetsu saponin IVa (CS); molecular weight is 794; molecular formula is C_42_H_66_O_14_. (**B**) The schematic diagram showing the timeline scheme of the animal experiments *in vivo*. (**C**) The levels of cholesterol and triglyceride in serum samples of mice fed with ND, HFD, HFD plus CS-L or HFD plus CS-H for 16 weeks (*n* = 10/group). (**D**) The levels of cholesterol and triglyceride in liver of mice fed with ND, HFD, HFD plus CS-L or HFD plus CS-H for 16 weeks (*n* = 10/group). All the data in (C–D) are mean ± standard deviation (SD); ^#^*p* < 0.01; *p < 0.05.

### CS treatment ameliorated HFD-induced inflammation in adipose tissue

Based on the aforementioned purpose, we determined the mRNA expression levels of several inflammation-related genes, including TNF-α, IL-6, MCP-1, CCL-5, CXCL-1 and SAA3, in epididymal adipose tissue (EAT). As shown in Figure 2A, compared with those of ND group, HFD could result in significant increases in mRNA expression levels of TNF-α, CCL-5, IL-6, CXCL-1, MCP-1 and SAA3 in EATs (*p* < 0.01); Treatment with Chikusetsu saponin IVa (CS-L and CS-H) caused significant inhibitions on the increased expression levels of these genes in EATs induced by HFD (*p* < 0.05) in a dose-dependent manner. However, while the fat weight of EAT was significantly higher in HFD than in ND group, the CS-L and CS-H treatments caused only slight but not significant reduction of the increased fat weights of EAT induced by HFD (Supplementary Figure 2).

**Figure 2:** CS treatment inhibits high fat diet-induced inflammation in adipose tissue (**A**) Real time PCR was used to detect the relative mRNA expression levels of TNF-α, MCP-1, IL-6, CCL-5, CXCL-1 and SAA3 in EAT from mice fed with ND, HFD, HFD plus CS-L or HFD plus CS-H for 16 weeks (*n* = 10/group). (**B**) The concentrations of TNF-α, MCP-1, IL-1β and Caspase-1 were determined in the supernatants of *ex vivo* cultured EAT isolated from mice fed with ND, HFD, HFD plus CS-L or HFD plus CS-H for 16 weeks (*n* = 10/group); Data in panels (A) and (B) are expressed as mean ± SD; ^#^*p* < 0.01, *p < 0.05.

To further determine whether these effects on mRNA expression levels of these genes could result in the corresponding alterations in the secretion of chemokines and cytokines, we isolated the EAT from mice fed with ND, HFD, HFD+CS-L or HFD+CS-H for 16 weeks, minced the EAT (0.8 g/mouse) and cultured them in DMEM medium without serum for 24 h. After culture for 24 h, their supernatants were harvested and the protein levels of TNF-α, MCP-1, IL-1β and Caspase-1 were measured with ELISA kits. Similar to what were observed at the mRNA expression levels, the concentrations of these proteins in the culture medium were significantly induced by HFD, which were all significantly decreased by CS-L and CS-H treatments in a dose-dependent manner (Figure 2B). Collectively, these data indicate that CS potently inhibits HFD-induced inflammation in adipose tissue.

### CS treatment inhibited the accumulation of adipose tissue macrophages (ATMs) and altered their polarization

ATMs have been known to play important roles in the formation of inflammation [3]. Based on the above described observations, we attempted to determine whether CS affects the infiltration of macrophages into adipose tissue. We examined the effects of CS on the mRNA expression levels of three macrophage markers, including CD11b, CD68, and F4/80. As shown in Figure 3A, the mRNA expression levels of CD11b, CD68, and F4/80 were increased significantly in EATs of HFD-fed mice, as compared with those of ND group, indicating that macrophages are actively recruited into adipose tissue by HFD. Consistent with its reduction of HFD-induced increases in mRNA expression levels of cytokines and chemokines, CS treatment significantly reduced the expression of these macrophage markers after 16 weeks of HFD (Figure 3A). We also observed a significant increase in the number of stromal vascular fraction (SVF) cells induced by HFD and the significant reductions in the number of SVF cells in EAT of mice treated with CS in a dose-dependent manner, as compared with those in HFD mice (Figure 3B). Furthermore, histological analysis also revealed much higher number of “crown-like structures” around adipocytes in HFD-fed mice than in ND mice, whereas numbers of “crown-like structures” were significantly reduced in CS-L and CS-H treated-HFD mice in a dose-dependent manner (Figure 3C), which were shown to represent the macrophages in fat tissues [20]. To further investigate the subset contents of these macrophages, we measured the mRNA expression levels of macrophage subtype-specific markers in EAT. The mRNA expression levels of two M1 macrophage markers, i.e. CD11c and iNOS, were increased significantly in HFD mice, as compared to those in ND mice. However, CS-L and CS-H treatments significantly decreased the mRNA expression levels of CD11c and iNOS in HFD mice (Figure 3D). In addition, the mRNA expression levels of two M2 macrophage markers, i.e. CD206 and Mgl2, were significantly reduced in HFD-fed mice as compared to those in ND mice while their mRNA expression levels were significantly increased in CS-L and CS-H treated HFD mice, as compared to those of HFD mice in a dose-dependent manner (Figure 3E). Collectively, these results indicate that CS treatment decreases the number of M1 macrophages but increases the number of M2 macrophages, therefore, decreasing the ratio of M1/M2 in EAT.

**Figure 3:** CS treatment inhibits the accumulation of ATMs and alters their polarization (**A**) Relative mRNA expression levels of macrophage markers in EAT from mice fed with ND, HFD, HFD plus CS-L or HFD plus CS-H for 16 weeks were determined by real time PCR (*n* = 10/group). (**B**) Cell number of SVF cells in EAT from mice fed with ND, HFD, HFD plus CS-L or HFD plus CS-H for 16 weeks (*n* = 10/group). (**C**) Representative images of H&E stained sections of EAT from mice fed with ND, HFD, HFD plus CS-L or HFD plus CS-H for 16 weeks (*n* = 10/group). Arrows head indicate the typical “crown-like structure (CLS)”. The scale bar is 50 μm. (**D**) Relative mRNA expression levels of M1 macrophage marker genes determined in EAT from mice fed with ND, HFD, HFD plus CS-L or HFD plus CS-H for 16 weeks (*n* = 10/group). (**E**) Relative mRNA expression levels of M2 macrophage marker genes determined in EAT from mice fed with ND, HFD, HFD plus CS-L or HFD plus CS-H for 16 weeks (*n* = 10/group). Data in panels A–E are expressed as mean ± SD; ^#^*p* < 0.01, *p < 0.05.

### CS treatment inhibited HFD-induced expression of NLRP3 inflammasome component genes and reduced NF-κB signaling in EAT

As shown in Figure 2B, CS treatment reduced HFD-induced secretion of both IL-1β and Caspase-1 in EAT culture supernatant. This observation prompted us to determine whether CS treatment affects the expression of NLRP3 inflammasome component genes, including IL-1, Caspase-1, Nlrp3, and Asc (Pycard) in EAT. Consistent with those reported previously [21], the mRNA expression levels of IL-1β, Caspase-1, Nlrp3, and Asc were all elevated in HFD-fed mice, as compared to those of ND mice (Figure 4A). CS-L and CS-H treatments significantly decreased the increased mRNA expression levels of these genes induced by HFD in a dose-dependent manner (Figure 4A). We also measured their protein expression levels in mice of these groups. Similar to the results of the mRNA expression levels of these genes, the protein expression levels of IL-1β, Caspase-1, Nlrp3, and Asc were also significantly increased in mice of HFD-fed groups, which were significantly reduced in mice of both CS-L and CS-H groups (Figure 4B). These data suggest that the anti-inflammatory effects of CS are likely mediated by inhibiting HFD-induced activation of NLRP3 inflammasome.

**Figure 4:** CS treatment inhibits HFD-induced expression levels of NLRP3 inflammasome component genes and reduces NF-κB signaling in EAT (**A**) Real time quantitative PCR was performed to measure the mRNA expression levels of NLRP3 inflammasome component genes in EAT from mice fed with ND, HFD, HFD plus CS-L or HFD plus CS-H for 16 weeks (*n* = 10/group). (**B**) Western blot analysis was performed to determine the protein expression levels of NLRP3 inflammasome components in EAT from mice fed with ND, HFD, HFD plus CS-L or HFD plus CS-H for 16 weeks. (**C**) Protein levels of NF-κB, IKK, IκB and their phosphorylated forms in EAT from mice fed with HFD, HFD plus CS-L or HFD plus CS-H for 16 weeks were measured by Western blot with corresponding antibodies (*n* = 10/group). Data are expressed as mean ± SD; ^#^*p* < 0.01, *p < 0.05. β-actin was used as the control for protein loading. The pictures are shown as the representative of at least three independent experiments.

In our previous study, we demonstrated that total saponin extracts from *Panax japonicus* (SPJ) and Chikusetsu saponin V, one main component of SPJ, could inhibit NF-κB signaling [18, 19]. Therefore, we determined whether CS could also have the inhibitory effects on NF-κB signaling by examining the levels of several important components of NF-κB signaling, including NF-κB, IKK, and IκB and their corresponding phosphorylated forms via Western blot analysis. As shown in Figure 4C and Supplementary Figure 3, while the total protein expression levels of NF-κB, IKK, and IκB were unchanged, their phosphorylated forms and the ratios of pNF-κB/NF-κB, pIKK/IKK, and pIκB/IκB were all decreased in EAT from HFD-fed mice treated with CS as compared with those of HFD mice. These results suggest that CS is also likely involved in inhibiting the HFD-induced activation of NF-κB signaling.

### CS potently inhibited ATP-induced activation of NLRP3 inflammasome in BMDMs

To further confirm whether CS-mediated inhibition of inflammation is via inhibition of NLRP3 inflammasome, BMDMs were treated with CS at the indicated concentrations for 24 h, stimulated with 1 μg/mL LPS for 4 h, and then exposed to 2 mM ATP for 1 h. The contents of IL-1β in culture supernatants were determined by ELISA. As shown in Figure 5A, neither LPS nor ATP alone caused much increased amounts of IL-1β, whereas their combination significantly induced IL-1β production. CS treatment could significantly inhibit IL-1β production induced by LPS plus ATP in a dose-dependent manner (Figure 5A). Meanwhile, CS treatment did not significantly affect the viability of BMDMs at the indicated concentrations (Supplementary Figure 4). Latz, E., *et al*. have reported that pro-IL-1β induction and caspase-1 activation are the important steps for IL-1β production induced by NLRP3[6]. To explore whether CS-mediated inhibition of LPS+ATP-induced IL-1β production is involved in these steps, we measured IL-1β protein level with western blot analyses. Consistent with the ELISA results (Figure 5A), LPS plus ATP induced IL-1β production and caspase-1 activation in BMDMs and increased extracellular secretion of IL-1β and caspase-1 (Figure 5B). As mentioned above, IL-1β production requires both priming and activating steps. We examined the effects of CS treatment on both steps. CS treatment significantly inhibited IL-1β production and caspase-1 activation induced by LPS plus ATP in BMDMs when CS was added at both priming and activating steps in a dose-dependent manner (Figure 5C). Pro-IL-1β expression was also decreased when BMDMs were treated with CS (Figure 5C). To further determine the effect of CS on inhibiting ATP-induced activation of NLRP3 inflammasome, we treated BMDMs with CS at either the priming or the activating step, respectively. As shown in Figure 5D, CS could inhibit pro-IL-1β expression induced by LPS when it was added at only the priming step but not at the activation step. Activation of caspase-1 was also inhibited by CS treatment, whereas IL-1β production was almost not inhibited (Figure 5D). However, caspase-1 expression and IL-1β production were remarkably reduced when CS was added at only the activating step (Figure 5E). Collectively, these data demonstrate that CS can inhibit ATP-induced activation of NLRP3 inflammasome.

**Figure 5:** CS inhibits the activation of NLRP3 inflammasome induced by ATP (**A**) BMDMs were treated with CS at the indicated concentrations for 24 h, and then stimulated with 1 μg/ml LPS for 4 h. The cells were washed twice with phosphate buffer saline (PBS), and finally exposed to 2 mM ATP for 1 h. The cells were also incubated with LPS, ATP, and medium alone. The supernatants were collected and IL-1β levels were determined by ELISA. The experiments were repeated at least three times independently, and the data are expressed as mean ± SD; ^#^*p* < 0.01, *p < 0.05 (*n* = 3). (**B**) BMDMs were stimulated with 0.2 μg/mL LPS for 4 h, and followed by incubating with 2 mM ATP for 1 h. The cells were also incubated with LPS, ATP and medium alone. After treatment, the culture supernatants and cell lysates were prepared, and western blot was performed with antibodies against caspase-1 and IL-1β in culture supernatants and cell lysates, respectively. (**C**–**E**) BMDMs were stimulated with 0.2 μg/ml LPS for 4 h, and followed by incubating with 2 mM ATP for 1 h. After being washed twice with PBS, the cells were subsequently treated with CS at the indicated concentrations for another 2 h, followed by stimulation with 0.2 μg/ml LPS for 16 h and 2 mM ATP for 6 h at the presence of CS at the indicated concentrations (C); or followed by stimulation with 0.2 μg/ml LPS for 22 h at the presence of CS at the indicated concentrations (D); or followed by stimulation with 2 mM ATP for 2 h at the presence of indicated concentrations of CS (E). From (C) to (E), the supernatants or cell lysates were prepared to perform Western blot analysis (the supernatants for caspase-1, IL-1β expression; the cell lysates for expression levels of pro-caspase-1, pro-IL-1β and β-actin, respectively). (**F**) BMDMs were treated with 20 μM CS, 10 μM parthenolide for 24 h, and then stimulated with 1 μg/mL LPS for 4 h, the cells were washed twice with PBS, and finally exposed to 2 mM ATP for 1 h at the presence of CS at the indicated concentrations or parthenolide. The supernatants or cell lysates were prepared to perform western blot analysis as mentioned above. The pictures in (B–F) are shown as the representative of three independent experiments.

Parthenolide derived from a plant has been reported to be a natural inhibitor of the NLRP3 inflammasome [22]. Thus, we compared the inhibitory effects of CS on inflammasome activation with those of parthenolide. Treatment of BMDMs with parthenolide remarkably decreased the expression levels of IL-1β and caspase-1 induced by ATP (Figure 5F). The inhibitory effects of CS were quite similar to those of parthenolide (Figure 5F).

### CS potently inhibited monosodium urate (MSU)-induced activation of NLRP3 inflammasome in BMDMs

MSU also engaged the NLRP3 inflammasome activation [23]. Thus, we attempted to determine whether CS can inhibit MSU-induced activation of NLRP3 inflammasome. As shown in Supplementary Figure 5A and 5B, LPS-induced slight increase in IL-1β but not caspase-1. MSU alone did not induce expression levels of IL-1β and caspase-1. LPS plus MSU substantially induced the activation of caspase-1 and IL-1β. CS potently inhibited caspase-1 activation and IL-1β production in BMDMs induced by MSU plus LPS.

On the other hand, in order to test the inhibitory effects of CS on IL-1β production in human cells, THP-1 cells, a human monocytic cell line, were firstly treated with 500 nM phorbol myristate acetate (PMA) for 3 h, and continuously cultured overnight without PMA to allow them to differentiate into macrophagic cells. As expected, CS inhibited LPS plus ATP- or LPS plus MSU-induced IL-1β production in these differentiated macrophages in a dose-dependent manner (Supplementary Figure 5C), suggesting that the inhibitory effects of CS on activation of NLRP3 inflammasome are not limited to mouse macrophages but also to human-derived cells such as THP-1 cells. Taken together, these results clearly demonstrate that CS is capable of inhibiting the activation of NLRP3 inflammasome induced by different stimuli.

### CS inhibited an NLRP3-induced formation of ASC pyroptosome and suppressesed the pyroptosis induced by LPS

The activation of NLRP3 inflammasome triggers the formation of ASC pyroptosome, which is a supramolecular assembly of ASC dimers involved in mediating inflammatory cell death via caspase-1 activation and is composed of ASC dimers [24]. As shown in Figure 6A, LPS plus ATP stimulation caused the formation of ASC dimers. However, parthenolide inhibited the formation of ASC pyroptosome induced by LPS plus ATP (Figure 6A). Similar to parthenolide, treatment of BMDMs with CS at 20 or 40 μM remarkably inhibited ASC pyroptosome formation induced by LPS plus ATP (Figure 6A). These data indicate that inhibition of activation of NLRP3 inflammasome may contribute to the inhibition of ASC pyroptosome.

**Figure 6:** CS inhibits the formation of NLRP3-induced ASC pyroptosome and pyroptosis (**A**) BMDMs were pretreated with 20 or 40 μM of CS, 10 μM of parthenolide for 24 h, and subsequently stimulated with 1 μg/mL of LPS for 4 h, followed by 2 mM of ATP for 1 h. The pellets cross-linked with disuccinimydyl suberate (DSS) and cell lysates were used for Western blot analysis with anti-ASC antibody. The concentrated supernatants (Supern) and cell lysates were used for Western blot analysis with anti-caspase-1 antibody. Pictures are the representative of three independent experiments. Panels (**B** and **C**) BMDMs were pretreated with CS at the indicated concentration for 24 h, and subsequently stimulated with 1 μg/ml of LPS for 4 h, followed by 2 mM of ATP for 1h, 2h, 4h, or 8h. Cell death was determined by measuring LDH release (B). The IL-1β levels in the supernatants were measured by ELISA (C). Data in (B) and (C) are shown as mean ± SD; ^#^*p* < 0.01, *p < 0.05.

Pyroptosis, a inflammatory form of programmed cell death, is dependent on caspase-1 and can be caused by inflammasome activation [25]. Pyroptotic cells destroy their structures and release lactate dehydrogenase (LDH), and also make macrophages easy to release IL-1β. To further confirm the effects of CS on the activation of NLRP3 inflammasome, we measured the LDH levels in BMDMs. As shown in Figure 6B, either LPS or ATP alone did not cause much release of LDH, LPS plus ATP stimulation caused an increasing release of LDH at 1, 2, 4 and 8 h in a time-dependent manner. CS significantly inhibited LDH release from BMDMs at 1, 2 and 4 h, but the inhibitory effects were not significant at 8 h after stimulation with LPS plus ATP. These suggest that CS can inhibit the pyroptosis. CS significantly inhibited LPS+ATP-induced expression of IL-1β from BMDMs at 1, 2, 4 and 8h (Figure 6C). However, the reduction of IL-1β release at 8 h after stimulation with LPS plus ATP was not mainly due to the suppression of pyroptosis (Figure 6C). Collectively, all of these data indicate that CS can inhibit the activation of NLRP3 inflammasome via inhibiting the pyroptosis.

### CS treatment inhibited the activation of NF-κB pathway in BMDMs induced by LPS

As mentioned above, we have found that CS can inhibit NF-κB activation in EAT of mice (Figure 4C and Supplementary Figure 3). To further confirm the inhibitory effect of CS on the NF-κB signaling, we treated BMDMs with CS at the indicated concentrations. As shown in Figure 7A, treatment of BMDMs with CS did not change the total protein levels of NF-κB p65 and IκB, but resulted in the significant decreases in levels of the phosphorylated forms of NF-κB p65 and IκB induced by LPS. Moreover, CS treatment significantly inhibited the nuclear DNA-binding ability of NF-κB (Figure 7B), strongly indicating the possibility that CS can inhibit the nuclear translocation of NF-κB. As expected, pretreatment of BMDMs with CS dose-dependently decreased the nuclear translocation of NF-κB p65 induced by LPS (Figure 7C). Furthermore, the LPS-induced mRNA expression levels of prostaglandin-endoperoxide synthase 2 (ptgs2) (Figure 7D) and nitrite oxide synthase-2 (NOS-2) (Figure 7F) were significantly inhibited by CS in BMDMs in a dose-dependent manner. Ptgs2 and NOS2 were the target genes of NF-κB [30]. CS significantly inhibited the TNF-α secretion stimulated by LPS in BMDMs in a dose-dependent manner (Figure 7F). Taken together, these data indicate that CS inhibits LPS-induced activation of NF-κB pathway and the expression of its target genes in BMDMs.

**Figure 7:** Effects of CS on LPS-induced NF-κB activation in BMDMs (**A**) After treatment with the indicated concentrations of CS for 24 h, BMDMs were stimulated with 1 μg/ml LPS for 4 h, cell lysates were prepared for western blot analysis with antibodies against NF-κB p65, phosphorylated NF-κB p65(pNF-κB p65), anti-IκB, and phosphorylated IκB(pIκB). (**B**) After treatment with CS at the indicated concentrations for 24 h, BMDMs were stimulated with 1 μg/mL LPS for 4 h. Nuclear extracts were prepared and subjected to EMSA. (**C**) After treatment with CS at the indicated concentrations for 24 h, BMDMs were stimulated with 1 μg/ml LPS for 4 h. Nuclear proteins were prepared for western blot analysis using anti-NF-κB p65 antibody. (**D**–**E**) BMDMs were treated as described above, the mRNA expression levels of ptgs2 and NOS2 were quantified by real time PCR. (**F**) The concentrations of TNF-α in the culture supernatants were measured by ELISA. All the data in (D–F) are expressed as mean ± SD; ^#^*p* < 0.01, *p < 0.05 (*n* = 3). All the pictures shown in (A–C) are the representative of at least three independent experiments.

## DISCUSSION

Obesity, including HFD-induced obesity, is associated with a number of chronic diseases such as triple negative breast cancer (TNBC) [26]. During the process of HFD-induced obesity, excessive fatty nutrition can induce the hypertrophic adipocytes, which play important roles in causing energy imbalance and dysregulation of metabolic pathways, and then adipocytes recruit macrophages into adipose tissues and secrete inflammatory cytokines and chemokines, thus, leading to formation of metabolic inflammation. There is a need of finding out medicines that can effectively ameliorate HFD-induced obesity.

In the present study, we demonstrated that CS could effectively ameliorate HFD-induced inflammation in adipose tissue, inhibit ATM accumulation and shift the polarization from M1 to M2. We also demonstrated an important role of CS in reducing production of pro-inflammatory cytokines, such as IL-1β, by suppressing the activation of NLRP3 inflammasome and NF-κB pathway induced by LPS, indicating that NLRP3 inflammasome and NF-κB pathway may be the important targets for CS anti-inflammatory activity.

Many pathological events, such as viral and bacterial infection and metabolic imbalance, can activate inflammasome. Among various inflammasomes, NLRP3 inflammasome has been associated with a number of human autoinflammatory and autoimmune diseases. NLRP3 inflammasome activation can finally result in chronic inflammation-associated diseases, such as insulin resistance, type-2 diabetes, obesity, and cancer etc. NLRP3 inflammasome may be a potentially important target for anti-inflammatory therapies [27]. Therefore, finding and identification of natural molecules capable of inhibiting NLRP3 inflammasome is of significance to develop effective therapeutics for inflammation-associated diseases.

Saponins from *Panax japonicus* (SPJ), the most abundant and active components in rhizoma of *Panax japonicus*, mainly include Panax saponins Re, Chikusetsu saponin V, Pjs-2, Chikusetsu saponin IV and Chikusetsu saponin IVa (CS) etc. [17]. We have demonstrated that SPJ and Chikusetsu saponin V, one component of SPJ, had anti-inflammatory and anti-oxidative activities [17–19, 28]. Herein, we demonstrated that CS, another major component of SPJ, also significantly improved HFD-induced lipid homeostasis and attenuated HFD-induced inflammation in adipose tissue of mice (Figure 1C–1D and Figure 2) as reflected by its inhibition of HFD-induced expression of pro-inflammatory cytokines (TNF-α and IL-6) and chemokines, including MCP-1, CCL-5, CXCL-1 and SAA3. It is worth noting that the same CS treatments did not significantly reduce the food intake and fat weight of EAT in mice (Supplementary Figures 1 and 2). The body weights of mice of HFD + CS-L and HFD + CS-H groups were slightly but not significantly decreased as compared with those in mice of HFD (data not shown), suggesting that treatments of mice with CS at the doses used and the intervention duration do not causes severe toxicity on the growth and development of EAT and body weight of mice. However, Li *et al*. [29] reported that CS treatment significantly decreased the body weight of rats. This is not consistent with our data, suggesting that the effects of CS on HFD-induced body weight in mice should be debated. This disparity may be related to differences in sources of CS, experimental animal strains (mice versus rats), drug doses and especially the intervention durations. Thus, the effects of CS on body weight in different animal strains, appropriate drug doses, the intervention duration and the toxicity *in vivo* need to be further investigated in more detail in our subsequent work for ensuring whether CS treatments at broader dose range and the entire duration during and after treatment can cause any significant toxicity.

Although white adipose tissues include visceral and subcutaneous adipose tissues, the former has greater capacity of macrophage recruitment and secrete more pro-inflammatory mediators than does the latter in responding to HFD [3]. Altintas *et al*. reported that macrophage infiltration into EAT was the most severe event in visceral adipose tissues [30]. Thus, we mainly focused on macrophages in EAT. The infiltration of ATM has been regarded as the important events during inflammation in adipose tissue [3]. We have proven that CS can ameliorate the HFD-induced inflammation in adipose tissue (Figure 2). Based this, we hypothesized that CS could suppress macrophage infiltration into adipose tissue. Our next experiments confirmed this hypothesis. As shown in Figure 3A–3C, CS attenuated macrophage infiltration into adipose tissues, decreased the number of M1 macrophages, increased the number of M2 macrophages, and shifted the ratio of M1/M2 in EATs as indicated by the decreased levels of M1-macrophage-specific markers and the increased levels of M2-macrophage-specific markers (Figure 3D–3E). CS can ameliorate obesity-associated inflammation in adipose tissue through potently inhibiting macrophage infiltration into adipose tissue. Macrophages are the important inflammatory cells and include 2 subtypes, namely M1 and M2 subtype. M1 subtype is mainly responsible for pro-inflammatory response while M2 subtype is mainly responsible for anti-inflammatory response. CS-induced reduction of M1 macrophages and the increase of M2 macrophages, and the reducted M1/M2 ratio further demonstrated that anti-inflammatory activity of CS is achieved, at least in part, through decreasing recruitment of M1 subpopulation and increasing recruitment of M2 subpopulation of macrophages.

M1 macrophages are the major sources of inflammatory cytokines such as TNF-α and IL-1β. They release cytokines via a series of orchestrated pathways, which are coordinated by multi-protein complexes. When being exposed to inflammatory stimuli, they secrete cytokines/chemokines e.g. TNF-α, IL-1, IL-6, IL-8, IL-12, as well as leukotrienes, prostaglandins, and complement. Together, these molecules enhance vascular permeability and recruitment of inflammatory cells and produce systemic effects such as the production of acute inflammatory response proteins and fever [31]. TNF-α stimulates the acute phase of the immune response and also exerts its effects in other organs [32]. For instance, it can stimulate the release of corticotropic releasing hormone, suppresses appetite, induces fever and stimulates the acute inflammatory response by enhancing the synthesis of C-reactive protein and other mediators in liver. It also induces vasodilation and loss of vascular permeability, which is propitious for lymphocyte, neutrophil, and monocyte infiltration and helps recruit these cells to the inflammation site by regulating chemokine release. In concord with IL-17, TNF-a can trigger the expression of neutrophil-attracting chemokine, e.g. CXCL-1, CXCL-2, and CXCL-5 [33] and augments the expression of cell adhesion molecules [34]. This, in turn, increases CXCL-2-dependent neutrophil migration to the inflammation site. Similarly to TNF-α, IL-1β is produced and released at the early stages of the immune response to infections, lesions, and stress. During inflammation, it stimulates the production of acute phase proteins from liver and acts on the central nervous system to induce fever and prostaglandin secretion. It also acts as a chemoattractant for granulocytes, enhances the differentiation of CD4 T cells [35], and increases the expression of cell adhesion molecules on leukocytes and endothelial cells. The inflammatory response is beneficial for the host when these cytokines are produced in appropriate amounts. However, they become toxic when being produced in a deregulated fashion. For instance, excess amounts of TNF-α play pathological roles in inflammatory-related diseases such as psoriasis, rheumatoid arthritis, asthma, cancer, infectious diseases, and other auto-immune pathologies. TNF-a and IL-1β released from activated (M1) macrophages might also contribute to NF-κB activation and form a vicious circle in promotion of inflammation (Figure 8).

**Figure 8:** Schematic illustration of CS-mediated inhibition of NLRP3 inflammasome and NF-κB signaling

M2 macrophages are further subdivided into M2a, M2b and M2c categories. M2a macrophages are involved in the Th2 type immune response. M2b macrophages are induced by IL-1, LPS and immune complexes and are involved in regulating immunity. They produce IL-10, IL-1, IL-6 and TNF-a. M2c macrophages are induced by IL-10 and TGF-β and regarded as deactivated or anti-inflammatory and participate in tissue repair and remodeling. They produce large amounts of IL-10 and TGF-β and express multiple receptors [36]. Thus, decreasing M1 macrophages and increasing M2 macrophages, and thus, significantly decreasing the ratio of M1/M2 in EAT by CS might disrupt and stop the vicious circle in promotion of inflammation. Base on the differentiation of macrophages, we will use BMDMs, the typical models for the studies on inflammation, to perform subsequent experiments for further elucidation of underlying mechanisms. In this study, we focused on macrophages. In the subsequent study, we need to investigate whether other types of immune/inflammatory cells are also involved in the anti-inflammatory effects of CS.

In this study, we clearly demonstrated that CS treatment inhibited HFD-induced expression of several key components (IL-1β, Caspase-1, Nlrp3 and Asc) of NLRP3 inflammasome at mRNA and protein level in EAT (Figure 4A and 4B). Moreover, CS treatment markedly inhibited HFD-induced caspase-1 and IL-1β production in EAT (Figure 2). Furthermore, we also found that CS inhibited ATP plus LPS- or MSU plus LPS-induced activation of NLRP3 inflammasome in BMDMs of mice or human THP-1 cells (Figure 5 and Supplementary Figure 5). Therefore, we propose that NLRP3 inflammasome is one of the important targets of CS for improving HFD-induced inflammation in adipose tissue. It is well accepted that priming signal is needed for the transcriptional regulation of NLRP3 inflammasome. In the present study, BMDMs were stimulated with LPS for 4 h at the priming step. It is a long duration of LPS stimulation. However, it has been suggested that fast stimulation of LPS (only 10 min) can prime the NLRP3 inflammasome [37, 38], which is regulated by mitochondria-derived reactive oxygen species (ROS). It was reported that ATP or MSU, which activated NLRP3 inflammasome, promoted ROS production, whereas scavengers of ROS blocked activation of NLRP3 inflammasome [39, 40]. Therefore, ROS has been inferred to act on the upstream of NLRP3 inflammasome. In future work, we will use fast LPS stimulation to determine whether CS can affect mitochondrial ROS production. NLRP3 inflammasome was recruited into mitochondria when it was activated [41]. Thus, future work is also required to investigate whether CS can affect the mitochondrial localization of NLRP3 in BMDMs when they are stimulated with LPS and/or ATP.

ASC forms large aggregates known as pyroptosome or “specks” when inflammasomes are activated [30]. Formation of ASC pyroptosome is involved in the activation of caspase-1 and processing of IL-1β. In this study, CS treatment inhibited the formation of ASC pyroptosome induced by LPS plus ATP in BMDMs (Figure 6A). Pyroptosis, a type of programmed cell death, can destroy cell structure and release LDH. We observed that CS treatment significantly inhibited LDH release from BMDMs induced by LPS plus ATP (Figure 6B). These are consistent with the reduction of ASC pyroptosome formation and IL-1β production.

NF-κB pathway is a prototypical proinflammatory signaling pathway, because NF-κB pathways are involved in regulating the expression of a large number of proinflammatory genes, such as cytokines, chemokines, and adhesion molecules [42]. In this study, we also found that CS treatment did not alter the protein levels of several key components of NF-κB pathway, including NF-κB, IKK, and IκB, but decreased the levels of their phosphorylated forms, and thus, the ratios of pNF-κB/NF-κB, pIKK/IKK, and pIκB/IκB in EAT of HFD-treated mice (Figure 4C and Figure 3). Our results indicated that CS could inhibit the NF-κB signaling, which is consistent with our previous results [18, 19]. It was reported that circulating LPS was increased in type-2 diabetic patients after a high fat meal [43, 44]. The experiments with animals also demonstrated that HFD increased circulating LPS [44]. Thus, it is likely that HFD could activate NF-κB signaling via LPS stimulation and that CS attenuated HFD-induced NF-κB activation might be involved in the inhibition of LPS stimulation. To confirm this possibility, we further used BMDMs to repeat these experiments, and found that CS inhibited LPS-induced NF-κB activation, nuclear translocation and expression of its target genes such as ptgs2, NOS2 and TNF-α (Figure 7).

We have shown that feeding mice with HFD significant increased the expression levels of inflammatory cytokines and chemokines including TNF-α, IL-1β, IL-6, CXCL-1, CCL-5, MCP-1 and SAA3 in EATs; Treatment with CS-L and CS-H significantly inhibited HFD-induced levels of these genes in EATs of HFD-fed mice in a dose-dependent manner. CS treatment reduced NF-κB signaling by significantly decreasing the phosphorylated forms and the ratios of pNF-κB/NF-κB, pIKK/IKK, and pIκB/IκB in EAT from HFD-fed mice as compared with those of HFD mice. These results suggest that CS is involved in reducing the activation of NF-κB signaling induced by HFD. In the resting state, inactive NF-κB dimer complexes are sequestered in cytoplasm due to the binding of inhibitory IκB proteins. Upon being stimulated by physiological and/or environmental stimulus, the IκB kinase (IKK) complex consisting of two catalytically active kinases (IKKα and IKKβ), is phosphorylated, which are then targeted for ubiquitination and proteasomal degradation, leading to the releases of the bound NF-κB dimers. The activated NF-κB dimers can translocate to the nucleus where they mediate transcriptional activation of a large number of down-stream genes [45]. NF-κB pathway is generally devised into the classical canonical and non-canonical NF-κB pathways [45]. In the canonical activation pathway, excitatory signaling is mediated via TNF receptor (TNFR), IL-1 receptor (IL-1R), Toll-like receptors (TLRs), and antigen receptors. TNFα, IL-1β, and LPS are typical stimulating signaling molecules [46, 47]. Stimulation via these receptors results in activation of IKK complex, which, in turn, phosphorylates IκBα primarily by IKK2. Thus, inhibition of NF-κB pathways by CS may be attributed to its suppression of HFD-induced expression of TNFα, IL-1β and other cytokines/chemokines. Thus, it is likely that the inhibition of NF-kB pathway by CS is mediated by down-regulation of TNF-α and IL-1β via the canonical NF-κB pathway. Non-canonical NF-κB activation requires coordinated assembly of a regulatory complex of the adaptors, including cIAP1, cIAP2, TRAF2 and TRAF3 and the kinase NIK [48] and is induced by TNF family cytokines, involves IKKα-mediated phosphorylation of p100 associated with RelB, leading to partial processing of p100 and the formation of transcriptionally active p52-RelB complexes. IKKα activation and phosphorylation of p100 depends on NIK, which is subject to complex regulation by TRAF3, TRAF2 and ubiquitin ligases. In this study, we did not investigate the effects of CS treatment on the expression levels of these adaptors and factors. Whether the inhibition of NF-κB pathways by CS is also mediated through non-canonical NF-κB pathway by inhibiting the expression and activities of these adaptors/factors remains to be determined.

Based on the findings made in this study, we concluded that CS could inhibit the adipose tissue inflammation via the mechanisms, which might be involved in suppressing the NLRP3 inflammasome activation and NF-κB signaling (Figure 8). It will also be inferred that CS can provide protective effects on many inflammatory diseases. NLRP3 inflammasome activation needs two steps which are involved in different mechanisms. The first step is the priming step in which NLRP3 transcription is induced; and the second step is posttranscriptional activation. NF-κB, the important mediator of inflammation, plays a critical role for the priming of NLRP3 inflammasome [49]. Thus, CS inhibits the NLRP3 priming through inhibiting NF-κB signaling, also via inhibiting the production of inflammatory cytokines such as TNF-α and IL-1β.

While this study was mainly focused on examining the effects of CS on inhibition of HFD-induced inflammation in adipose tissue, we also found that CS conferred similar inhibitory effects on inflammation in human THP-1 cells and on inflammations induced by LPS plus ATP- and MSU plus ATP-induced formation of NLRP3 inflammasome. These findings suggest that CS can confer anti-inflammatory effects in other organs/tissues and other diseases including cancer. It has been reported that activation of NLRP3 inflammasome enhanced the proliferation and migration of A549 lung cancer cells [50] and that obesity-associated NLRC4 inflammasome activation/IL-1 signaling promoted breast cancer progression [51]. Obesity has been linked to an increased risk of developing breast cancer and worse clinical prognosis [52] and is a risk factor for TNBC [26]. Within the tumor microenvironment in the context of obesity, an increase in tumor-infiltrating myeloid cells is induced with an activated NLRC4 inflammasome, which, in turn, activates IL-1β, driving disease progression through enhancing the expression of adipocyte-mediated vascular endothelial growth factor A and angiogenesis. In mice treated with metformin, obesity-associated tumor progression was inhibited and associated with a marked decrease in angiogenesis [51], suggesting a useful basis for treatment of patients with obese-related cancer by blocking NLRC4 inflammasome activation and/or IL-1β signaling transduction. Thus, CS and other main components of SPJR, including Chikusetsu saponin V, Chikusetsu saponin IV, Panax saponins Re, and Pjs-2, can be explored to block activation of NLRC4 inflammasome and/or IL-1β signaling transduction in patients with obese-related cancer and TNBC. This possibility merits further exploration.

## MATERIALS AND METHODS

### Reagents

Chikusetsu saponin IVa (CS) was originally isolated from total saponins of *Panax japonicus* collected from Enshi Chunmuying Medicinal Materials Planting Base, and identified by professor Kun Zou. CS (purity > 98%) was finally purchased from Chengdu Purechem-Standard Co., Ltd (Chengdu, Sichuan, China). The specimen was maintained in Hubei Key Laboratory of Natural Products Research and Development in China Three Gorges University. The chemical structure of CS was shown in Figure1A. ATP, lipopolysaccharide(LPS)(055:B5) and parthenolide were obtained from Sigma-Aldrich (St. Louis, MO, USA). Monosodium urate (MSU) was obtained from Enzo Life Sciences (NY, USA). Primary antibodies against phospho-IκB and Asc were obtained from Santa Cruz Biotechnology (Santa Cruz, CA, USA). Antibodies against Caspase-1, phospho-IKKα/β (Ser176/180), IKKα, phospho-NFκB p65(Ser536) and NFκB p65 were purchased from Cell Signaling Technology (Danvers, MA, USA). Antibodies for IL-1β and NLRP3 were purchased from abcam (Cambridge, UK). The food for the mice was purchased from Beijing HFK Bioscience CO. LTD(Beijing, China). Other reagents were obtained from Sigma-Aldrich.

### Experimental mice and protocol

Male C57BL/6 mice (4-week old, 18–22 g) were obtained from Chongqing Medical University (Chongqing, China) with quality certificated number SYXK 2007-0001. The mice were kept under pathogen-free conditions, and had free access to water and food. The experiments were performed according to the guidelines for the Ethics Committee Guide of China Three Gorges University after the mice were acclimated for one week.

The experimental protocols with mice were schematically illustrated in Figure 1B. The mice were randomly divided into four groups with 10 mice per group, fed and treated as follows: normal diet (ND) containing 10% fat; HFD containing 60% fat; HFD + CS-L (50 mg/kg of CS) and HFD + CS-H (100 mg/kg of CS). CS was given by gavage. For control, the mice in ND and HFD groups were given 0.9% sodium chloride by gavage. The treatments were maintained for 16 weeks (Figure 1B). During this period, the water intake and food consumption were measured and recorded daily while body weight was monitored weekly. At the end of treatment, the mice were euthanized using CO_2_ inhalation, and their serum and liver samples were collected. The levels of total cholesterol and triglyceride in serum and liver were measured by the commercial kits according to the protocols (Roche Diagnostics, Mannheim, Germany). The epididymal adipose tissue (EAT) was isolated, weighted and stored at −80°C for further analysis.

### Morphological observations

The EATs isolated from the experimental mice were fixed in 4% formaldehyde solution for at least 24 h, and embedded in paraffin. 5-μm serial sections were cut, and then stained with hematoxylin and eosin (HE).

### *Ex vivo* culture of EATs

The EATs isolated from the experimental mice were minced into small pieces and seeded into 24-well plates (0.8g/mouse) with serum-free DMEM medium, supplemented with 2 mM L-glutamine, 100 units/mL penicillin and 100 mg/mL streptomycin. After culture at 37°C under 5% CO_2_ for 24 h, the supernatants were harvested. The levels of TNF-α, MCP-1, IL-1β and caspase-1 in the supernatants were determined using corresponding commercial ELISA kits.

### Culture and stimulation of mouse bone marrow derived macrophages (BMDMs) and human THP-1 cells

BMDMs were isolated from C57BL/6 mice and seeded in 10-cm dishes with DMEM medium supplemented with 10% fetal bovine serum (FBS) and 100 ng/ml colony stimulating factor (CSF) at 37°C under 5% CO_2_. After culture for 6 days, the adherent cells were collected and served as BMDMs. They were stimulated with LPS at 0.2 μg/mL or 1 μg/mL as described previously [11, 53].

Human THP-1 cell line was initially obtained from American Type Culture Collection (ATCC, Manassas, VA, USA). After being treated with 500 nM phorbol myristate acetate (PMA) for 3 h, and washed twice with PBS, human THP-1 cells were cultured overnight without PMA to differentiate them into macrophagic cells.

### Real-time PCR

The extraction of total RNA and cDNA synthesis were performed as described in our previous studies [54, 55]. SYBR Green Master Mix kit (Qiagen, Netherlands) was used to perform real time PCR. The amplification program was performed as follows: pre-incubation at 50°C, 2 min; denaturation at 95°C, 10 min; followed by subsequently by 40 cycles of 95°C, 15 sec; and 60°C, 60 sec. The mRNA expression level was calculated by 2^−ΔΔCt^ method, using GAPDH as the endogenous control. The PCR primers were listed in Supplementary Table 1 in the Supplementary materials.

### Western blot analysis

Protein extraction from the tissues of mice or the treated cells and its concentration measurement were performed as described in previous studies [55, 56]. Denatured protein samples (50 μg/lane) were fractionated in 4–15% sodium dodecyl sulfate polyacrylamide gel electrophoresis (SDS-PAGE) gel and transferred to polyvinylidene difluoride (PVDF) membrane. The membrane was blocked with 5% milk for 1 h, then incubated with the indicated primary antibodies specific to the target proteins overnight, and finally incubated with one of the corresponding specific secondary antibodies for 1 hr. Antibody for β-actin was served as the control. The proteins bound by the specific antibody were detected using ECL Super Signal reagent (Pierce, Rockford, IL, USA) and exposed to the X-ray film for autoradiography.

### Isolation of stromal vascular fraction (SVF) cells

Isolation of SVF cells was conducted following the previously published method [57] with slight modifications. Briefly, EATs were isolated from mice fed with ND, HFD, HFD plus CS-L or HFD plus CS-H, weighed and rinsed with PBS. The minced adipose tissue was digested with Krebs-Ringer bicarbonate (KRB) buffer containing 280 U/mL collagenase I at 37°C for 30 min and then filtered through a 40-μm mesh. SVF cells were obtained after centrifugation at 600 g for 5 min. The SVF cells were stained with PE or FITC conjugated anti-mouse antibodies against CD11b, CD68, and F4/80, and then analyzed by flow cytometer (Becton-Dickinson, Franklin Lakes, NJ, USA).

### Measurement of lactate dehydrogenase (LDH) release

BMDMs were pretreated with CS at the indicated concentrations for 24 h, and subsequently stimulated with LPS at 1 μg/ml for 4 h, followed by treatment with 2 mM ATP for 1, 2, 4, or 8 h, respectively. The supernatants were collected and analyzed for LDH release using the Homogeneous Membrane Integrity Assay (Promega, Madison, WI, USA) according to the manufacturer's instructions.

### Electrophoretic mobility shift assay (EMSA)

The extraction of nuclear protein was performed following the commercial nuclear protein extraction kit (Bayotime, Shanghai, China), and the protein level was measured by Bradford method. The interaction between CS and NF-κB was determined using Chemiluminescent EMSA Kit (Rockford, IL, USA). Briefly, ^32^P-labeled NF-κB oligonucleotide (5′-GTTCGACAGAGGGGACTT

TCCGAGAGGCAAC-3′) was incubated with equal nuclear extract for 20 min. Each binding reaction system was separated in 4% polyacrylamide gel, and transferred onto the pre-soaked nylon membranes. The cross-linking between the transferred DNA and membranes was performed using a UV light cross-linker instrument. The membranes were then blocked with blocking buffer for 15 min and finally analyzed by autoradiography.

### Statistical analysis

The data obtained from three independently repeated experiments were presented as mean ± SD. Statistical analyses were performed using Student's *t-test* or one-way ANOVA analysis following Bonferroni *post hoc* with SPSS 18.0 software. *P* < 0.05 was set for statistical significance.

## SUPPLEMENTARY MATERIALS FIGURES AND TABLES


